The article "A Comprehensive Review on Metabolic Syndrome" was retracted in 2019. Reasons: plagiarism; overlap with other authors' work.

# A Comprehensive Review on Metabolic Syndrome

**DOI:** 10.1155/2014/943162

**Published:** 2014-03-11

**Authors:** Jaspinder Kaur

**Affiliations:** Ex-Servicemen Contributory Health Scheme (ECHS) Polyclinic, Sultanpur Lodhi, Kapurthala District 144626, India

## Abstract

Metabolic syndrome is defined by a constellation of interconnected physiological, biochemical, clinical, and metabolic factors that directly increases the risk of cardiovascular disease, type 2 diabetes mellitus, and all cause mortality. Insulin resistance, visceral adiposity, atherogenic dyslipidemia, endothelial dysfunction, genetic susceptibility, elevated blood pressure, hypercoagulable state, and chronic stress are the several factors which constitute the syndrome. Chronic inflammation is known to be associated with visceral obesity and insulin resistance which is characterized by production of abnormal adipocytokines such as tumor necrosis factor **α**, interleukin-1 (IL-1), IL-6, leptin, and adiponectin. The interaction between components of the clinical phenotype of the syndrome with its biological phenotype (insulin resistance, dyslipidemia, etc.) contributes to the development of a proinflammatory state and further a chronic, subclinical vascular inflammation which modulates and results in atherosclerotic processes. Lifestyle modification remains the initial intervention of choice for such population. Modern lifestyle modification therapy combines specific recommendations on diet and exercise with behavioural strategies. Pharmacological treatment should be considered for those whose risk factors are not adequately reduced with lifestyle changes. This review provides summary of literature related to the syndrome's definition, epidemiology, underlying pathogenesis, and treatment approaches of each of the risk factors comprising metabolic syndrome.

## 1. Introduction

The metabolic syndrome (MetS) is a major and escalating public-health and clinical challenge worldwide in the wake of urbanization, surplus energy intake, increasing obesity, and sedentary life habits. MetS confers a 5-fold increase in the risk of type 2 diabetes mellitus (T2DM) and 2-fold the risk of developing cardiovascular disease (CVD) over the next 5 to 10 years [1]. Further, patients with the MetS are at 2- to 4-fold increased risk of stroke, a 3- to 4-fold increased risk of myocardial infarction (MI), and 2-fold the risk of dying from such an event compared with those without the syndrome [2] regardless of a previous history of cardiovascular events [3]. A version of MetS has a WHO International Classification of Disease (ICD-9) code (277.7) which permits healthcare reimbursement. This shows that the term “metabolic syndrome” is institutionalized and a part of the medical vocabulary. MetS is considered as a first order risk factor for atherothrombotic complications. Its presence or absence should therefore be considered an indicator of long-term risk. On the other hand, the short-term (5–10 years) risk is better calculated using the classical algorithms (Framingham, REGICOR {Registre GIroní del COR}), as they include age, sex, total cholesterol or LDL, and smoking [4].

The article "A Comprehensive Review on Metabolic Syndrome" was retracted in 2019. Reasons: plagiarism; overlap with other authors' work.

## 2. Background

MetS started as a concept rather than a diagnosis [11]. The metabolic syndrome has its origins in 1920 when Kylin, a Swedish physician, demonstrated the association of high blood pressure (hypertension), high blood glucose (hyperglycemia), and gout [12]. Later in 1947, Vague described that the visceral obesity was commonly associated with the metabolic abnormalities found in CVD and T2DM [13]. Following this, in 1965, an abstract was presented at the European Association for the Study of Diabetes annual meeting by Avogaro and Crepaldi [14] which again described a syndrome which comprised hypertension, hyperglycemia, and obesity. The field moved forward significantly following the 1988 Banting Lecture given by Reaven [15]. He described “a cluster of risk factors for diabetes and cardiovascular disease” and named it “Syndrome X”. His main contribution was an introduction of the concept of the insulin resistance. However, he surprisingly missed obesity or visceral obesity from the definition which was later added as a crucial abnormality. In 1989, Kaplan [16] renamed the syndrome “The Deadly Quartet” for the combination of upper body obesity, glucose intolerance, hypertriglyceridemia, and hypertension and however, in 1992, it was again renamed “The Insulin Resistance Syndrome” [17]. Several groups have attempted to develop diagnostic criteria for the diagnosis of the MetS [18]. The first attempt was made by a World Health Organization (WHO) diabetes group in 1998 to provide a definition of the MetS [5]. In response, the European Group for the study of Insulin Resistance (EGIR) countered with a modification of the WHO definition in 1999 [6]. In 2001, the National Cholesterol Education Program Adult Treatment Panel (NCEP/ATP) released its definition [7]. Subsequently, the American Association of Clinical Endocrinologists (AACE) in 2003 offered its views regarding the definition of the syndrome [8]. The proliferation of definitions suggested that a single unifying definition was desirable [19]. In the hope of accomplishing this, the International Diabetes Federation (IDF) proposed a new definition of the MetS in April 2005 [9].

## 3. Definition

MetS is defined by a constellation of an interconnected physiological, biochemical, clinical, and metabolic factors that directly increases the risk of atherosclerotic cardiovascular disease (ASCVD), (T2DM), and all cause mortality [20, 21]. This collection of unhealthy body measurements and abnormal laboratory test results include atherogenic dyslipidemia, hypertension, glucose intolerance, proinflammatory state, and a prothrombotic state. There have been several definitions of MetS, but the most commonly used criteria for definition at present are from the World Health Organization (WHO) [5], the European Group for the study of Insulin Resistance (EGIR) [6], the National Cholesterol Education Programme Adult Treatment Panel III (NCEP ATP III) [7], American Association of Clinical Endocrinologists (AACE) [8], and the International Diabetes Federation (IDF) [9] (Table 1).

The article "A Comprehensive Review on Metabolic Syndrome" was retracted in 2019. Reasons: plagiarism; overlap with other authors' work.

Although each definition possesses common features, there are several parameters that differ which results in difficulty in terms of applicability, uniformity, and positive predictive value with all these definitions. The AACE, WHO, and EGIR definitions are all largely focused on insulin resistance, which is determined by an oral glucose tolerance test and hyperinsulinemic-euglycemic clamp. However, this labour intensive method is primarily used in a research environment [22]. In contrast, the ATPIII definitions were developed which use measurements and laboratory results that are readily available to physicians, facilitating their clinical and epidemiological application and therefore have remained a backbone for subsequent classifications such as the IDF diagnostic criterion [22]. However, a major problem with the WHO and NCEP ATP III definitions has been their applicability to the different ethnic groups, especially when trying to define obesity cut-offs. This is particularly evident for the risk of T2DM, which is apparent at much lower levels of obesity in Asians compared to Europeans. The IDF, having recognized the difficulties in identifying unified criteria for MetS that were applicable across all the ethnicities, has proposed a new set of criteria with ethnic/racial specific cut-offs [1] (Table 2). This accounts for the fact that the different populations, ethnicities, and nationalities have the different distributions of norms for body weight and waist circumference. It also recognizes that the relationship between these values and the risk of T2DM or CVD differs in different populations.

## 4. Epidemiology

Worldwide prevalence of MetS ranges from <10% to as much as 84%, depending on the region, urban or rural environment, composition (sex, age, race, and ethnicity) of the population studied, and the definition of the syndrome used [23, 24]. In general, the IDF estimates that one-quarter of the world's adult population has the MetS [9]. Higher socioeconomic status, sedentary lifestyle, and high body mass index (BMI) were significantly associated with MetS. Cameron et al. have concluded that the differences in genetic background, diet, levels of physical activity, smoking, family history of diabetes, and education all influence the prevalence of the MetS and its components [25]. The observed prevalence of the MetS in National Health and Nutrition Examination Survey (NHANES) was 5% among the subjects of normal weight, 22% among the overweight, and 60% among the obese [26]. It further increases with age (10% in individuals aged 20–29, 20% in individuals aged 40–49, and 45% in individuals aged 60–69) [27]. The prevalence of MetS (based on NCEP-ATP III criteria, 2001) varied from 8% to 43% in men and from 7% to 56% in women around the world [25]. Park et al. [26] noticed that there is an increase in the prevalence of MetS from 20 years old through the sixth and seventh decade of life for males and females, respectively. Ponholzer et al. reported that there is high prevalence of MetS among postmenopausal women, which varies from 32.6% to 41.5% [28]. A Framingham Heart Study report indicated that a weight increase of ≥2.25 kg over a period of 16 yr was associated with an up to 45% increased risk of developing the MetS [29], and it has been shown by Palaniappan et al. that each 11 cm increase in waist circumference (WC) is associated with an adjusted 80% increased risk of developing the syndrome within 5 years [30]. The metabolic alterations occur simultaneously more frequently than would be expected by chance and the concurrence of several factors increases cardiovascular risk over and above the risk associated with the individual factors alone [31]. The risk increases with the number of MetS components present [32].

The article "A Comprehensive Review on Metabolic Syndrome" was retracted in 2019. Reasons: plagiarism; overlap with other authors' work.

## 5. Pathophysiology

MetS is a state of chronic low grade inflammation as a consequence of complex interplay between genetic and environmental factors. Insulin resistance, visceral adiposity, atherogenic dyslipidemia, endothelial dysfunction, genetic susceptibility, elevated blood pressure, hypercoagulable state, and chronic stress are the several factors which constitute the syndrome (Figure 1).

### 5.1. Abdominal Obesity

The “obesity epidemic” is principally driven by an increased consumption of cheap, calorie-dense food and reduced physical activity. Adipose tissue is a heterogeneous mix of adipocytes, stromal preadipocytes, immune cells, and endothelium, and it can respond rapidly and dynamically to alterations in nutrient excess through adipocytes hypertrophy and hyperplasia [33]. With obesity and progressive adipocytes enlargement, the blood supply to adipocytes may be reduced with consequent hypoxia [34]. Hypoxia has been proposed to be an inciting etiology of necrosis and macrophage infiltration into adipose tissue that leads to an overproduction of biologically active metabolites known as adipocytokines which includes glycerol, free fatty acids (FFA), proinflammatory mediators (tumor necrosis factor alpha (TNF*α*) and interleukin-6 (IL-6)), plasminogen activator inhibitor-1 (PAI-1), and C-reactive protein (CRP) [35]. This results in a localized inflammation in adipose tissue that propagates an overall systemic inflammation associated with the development of obesity related comorbidities [36]. Adipocytokines integrate the endocrine, autocrine, and paracrine signals to mediate the multiple processes including insulin sensitivity [37], oxidant stress [38], energy metabolism, blood coagulation, and inflammatory responses [39] which are thought to accelerate atherosclerosis, plaque rupture, and atherothrombosis. This shows that the adipose tissue is not only specialized in the storageand mobilization of lipids but it is also a remarkable endocrine organ releasing the numerous cytokines.

#### 5.1.1. FFA

Upper body subcutaneous adipocytes generate a majority of circulating FFA while an intra-abdominal fat content has been positively correlated with the splanchnic FFA levels which may contribute to the liver fat accumulation commonly found in abdominal obesity [40]. Further, an acute exposure of skeletal muscle to the elevated levels of FFA induces insulin resistance by inhibiting the insulin-mediated glucose uptake, while, a chronic exposure of the pancreas to the elevated FFA impairs a pancreatic *β*-cell function [41]. FFAs increase fibrinogen and PAI-1 production [42].

#### 5.1.2. TNF*α*

It is a paracrine mediator in adipocytes and appears to act locally to reduce the insulin sensitivity of adipocytes [35]. Evidence suggests that TNF-**α** induces adipocytes apoptosis [43] and promotes insulin resistance by the inhibition of the insulin receptor substrate 1 signalling pathway [44]. The paracrine action would further tend to exacerbate the FFA release, inducing an atherogenic dyslipidemia [45]. Plasma TNF*α* is positively associated with the body weight, WC, and triglycerides (TGs), while, a negative association exists between the plasma TNF*α* and High density lipoprotein–cholesterol (HDL-C) [43].

#### 5.1.3. CRP

Elevated levels of CRP are associated with an increased WC [46], insulin resistance [47], BMI [48], and hyperglycemia [46] and are increased with the number of the MetS components. It is more likely to be elevated in obese insulin-resistant, but, not in obese insulin-sensitive subjects [49]. In addition, it has been demonstrated that regardless of the presence or degree of the MetS in an individual, CRP levels independently predicted the occurrence of future CVD events [50]. Because the MetS has been linked with a greater chance of future CVD events [51], CRP levels may be an important independent predictor of unfavourable outcomes in the MetS.

The article "A Comprehensive Review on Metabolic Syndrome" was retracted in 2019. Reasons: plagiarism; overlap with other authors' work.

#### 5.1.4. IL-6

It is released by both adipose tissue and skeletal muscle in humans [52]. It has both an inflammatory and an anti-inflammatory action. IL-6 receptor is also expressed in the several regions of the brain, such as the hypothalamus, in which it controls an appetite and energy intake [53]. It is a systemic adipokine, which not only impairs insulin sensitivity but is also a major determinant of the hepatic production of CRP [54]. IL-6 is capable of suppressing lipoprotein lipase activity. It has been shown to be positively associated with BMI, fasting insulin, and the development of T2DM [55] and negatively associated with HDL-C [56].

#### 5.1.5. PAI-1

A serine protease inhibitor is secreted from intra-abdominal adipocytes, platelets, and the vascular endothelium [35]. It exerts its effects by inhibiting the tissue plasminogen activator (tPA) [57] and thus is considered as a marker of an impaired fibrinolysis and atherothrombosis. Plasma PAI-1 levels are increased in abdominally obese subjects [58] and inflammatory states [59], thus, increasing the risk of an intravascular thrombus and adverse cardiovascular outcomes [60].

#### 5.1.6. Adiponectin

It regulates the lipid and glucose metabolism, increases insulin sensitivity, regulates food intake and body weight, and protects against a chronic inflammation [61]. It inhibits hepatic gluconeogenic enzymes and the rate of an endogenous glucose production in the liver. It increases glucose transport in muscles and enhances fatty acid oxidation [18]. It has a multifactorial antiatherogenic action which includes an inhibition of endothelial activation, a reduced conversion of macrophages to foam cells, and inhibition of the smooth muscle proliferation and arterial remodelling that characterizes the development of the mature atherosclerotic plaque [62]. Adiponectin is inversely associated with CVD risk factors such as blood pressure, low density lipoprotein cholesterol (LDL-C), and TGs [63]. Moreover, Pischon et al. have shown adiponectin to be a strong inverse independent risk factor for CVD [64]. Further, Fumeron et al. concluded that hypoadiponectinemia is associated with insulin resistance, hyperinsulinemia, and the possibility of developing T2DM, independent of fat mass [65]. The anti-inflammatory molecule, adiponectin, is negatively associated with the body weight, WC, TGs, fasting insulin, insulin resistance (HOMA-Homeostasis Model Assessment) [43], BMI, and blood pressure, whereas a positive association exists between adiponectin and HDL-C [43, 66]. Its expressions and secretions are reduced by TNF*α* [67], possibly through a stimulated production of IL-6, which also inhibits adiponectin secretion [68]. Adiponectin is seen to be “protective,” not only in its inverse relationship with the features of MetS [69] but also through its antagonism of TNF*α* action [70].

The article "A Comprehensive Review on Metabolic Syndrome" was retracted in 2019. Reasons: plagiarism; overlap with other authors' work.

#### 5.1.7. Leptin

It is an adipokine involved in the regulation of satiety and energy intake [35]. Levels of leptin in the plasma increase during the development of obesity and decline during the weight loss. Leptin receptors are located mostly in the hypothalamus and the brain stem and signals through these receptors controls satiety, energy expenditure, and neuroendocrine function. Most overweight and obese individuals have an elevated level of leptin that do not suppress appetite, or in other words, leptin resistance. Leptin resistance is thought to be a fundamental pathology in obesity [71]. Besides its effect on appetite and metabolism, leptin acts in the hypothalamus to increase the blood pressure through activation of the sympathetic nervous system (SNS) [72]. High circulating levels of leptin are reported to explain much of the increase in the renal sympathetic tone observed in obese human subjects [73]. Leptin-induced increase in renal sympathetic activity and blood pressure is mediated by the ventromedial and dorsomedial hypothalamus [74]. Leptin is an nitric oxide (NO) dependent vasodilator but also increases the peripheral vascular resistance and the sympathetic nerve activity [75]. The concentration of plasma leptin is correlated with adiposity, and hyperleptinemia is indeed considered an independent cardiovascular disease risk factor [76].

### 5.2. Insulin Resistance

Characteristics of the insulin-sensitive phenotype include a normal body weight [77] without abdominal or visceral obesity [78], being moderately active [79], and consuming a diet low in saturated fats [80]. Alternatively, insulin-resistant individuals demonstrate an impaired glucose metabolism or tolerance by an abnormal response to a glucose challenge, an elevated fasting glucose levels and/or overt hyperglycemia, or a reduction in insulin action after intravenous administration of insulin (euglycemic clamp technique) with decreased insulin-mediated glucose clearance and/or reductions in the suppression of endogenous glucose production. It is defined as a pathophysiological condition in which a normal insulin concentration does not adequately produce a normal insulin response in the peripheral target tissues such as adipose, muscle, and liver. Under this condition, pancreatic beta cell secretes more insulin (i.e., hyperinsulinemia) to overcome the hyperglycemia among insulin-resistant individuals. Although hyperinsulinemia may compensate for insulin resistance to some biological actions of insulin, that is, maintenance of normoglycemia, however, it may cause an overexpression of insulin activity in some normally sensitive tissues. This accentuation of some insulin actions coupled with a resistance to other actions of insulin results in the clinical manifestations of MetS [81]. An inability of the pancreatic beta cells over time to produce a sufficient insulin to correct the worsening tissue insulin resistance leads to hyperglycemia and overt T2DM [82]. Physiological insulin signalling occurs following the binding of insulin to the insulin receptor, a ligand-activated tyrosine kinase. Binding of insulin results in a tyrosine phosphorylation of downstream substrates and activation of two parallel pathways: the phosphoinositide 3-kinase (PI3K) pathway and the mitogen activated protein (MAP) kinase pathway. The PI3K-Akt pathway is affected, while, the MAP kinase pathway functions normally in insulin resistance. This leads to a change in the balance between these two parallel pathways. Inhibition of the PI3K-Akt pathway leads to a reduction in endothelial NO production, resulting in an endothelial dysfunction, and a reduction in GLUT4 translocation, leading to a decreased skeletal muscle and fat glucose uptake. By contrast, the MAP kinase pathway is unaffected, so there is a continued endothelin-1 (ET-1) production, an expression of vascular cell adhesion molecules, and a mitogenic stimulus to vascular smooth muscle cells. In these ways, an insulin resistance leads to the vascular abnormalities that predispose to atherosclerosis. Although insulin-resistant individuals need not be clinically obese, they nevertheless commonly have an abnormal fat distribution that is characterized by a predominant upper body fat. Regardless of the relative contributions of visceral fat and abdominal subcutaneous fat to insulin resistance, a pattern of abdominal (or upper body) obesity correlates more strongly with the insulin resistance and the MetS than does lower body obesity [83].

The article "A Comprehensive Review on Metabolic Syndrome" was retracted in 2019. Reasons: plagiarism; overlap with other authors' work.

### 5.3. Dyslipidemia

This dyslipidemia is characterised by a spectrum of qualitative lipid abnormalities reflecting perturbations in the structure, metabolism, and biological activities of both atherogenic lipoproteins and antiatherogenic HDL-C which includes an elevation of lipoproteins containing apolipoprotein B (apoB), elevated TGs, increased levels of small particles of LDL, and low levels of HDL-C. Insulin resistance leads to an atherogenic dyslipidemia in several ways. First, insulin normally suppresses lipolysis in adipocytes, so an impaired insulin signalling increases lipolysis, resulting in increased FFA levels. In the liver, FFAs serve as a substrate for the synthesis of TGs. FFAs also stabilize the production of apoB, the major lipoprotein of very low density lipoprotein (VLDL) particles, resulting in a more VLDL production. Second, insulin normally degrades apoB through PI3K-dependent pathways, so an insulin resistance directly increases VLDL production. Third, insulin regulates the activity of lipoprotein lipase, the rate-limiting and major mediator of VLDL clearance. Thus, hypertriglyceridemia in insulin resistance is the result of both an increase in VLDL production and a decrease in VLDL clearance. VLDL is metabolized to remnant lipoproteins and small dense LDL, both of which can promote an atheroma formation. The TGs in VLDL are transferred to HDL by the cholesterol ester transport protein (CETP) in exchange for cholesteryl esters, resulting in the TG-enriched HDL and cholesteryl ester-enriched VLDL particles. Further, the TG-enriched HDL is a better substrate for hepatic lipase, so it is cleared rapidly from the circulation, leaving a fewer HDL particles to participate in a reverse cholesterol transport from the vasculature. Thus, in the liver of insulin-resistant patients, FFA flux is high, TGs synthesis and storage are increased, and excess TG is secreted as VLDL [84]. For the most part, it is believed that the dyslipidemia associated with insulin resistance is a direct consequence of increased VLDL secretion by the liver [85]. These anomalies are closely associated with an increased oxidative stress and an endothelial dysfunction, thereby reinforcing the proinflammatory nature of macrovascular atherosclerotic disease.

### 5.4. Hypertension

Essential hypertension is frequently associated with the several metabolic abnormalities, of which obesity, glucose intolerance, and dyslipidemia are the most common [86]. Studies suggest that both hyperglycemia and hyperinsulinemia activate the Renin angiotensin system (RAS) by increasing the expression of angiotensinogen, Angiotensin II (AT II), and the AT1 receptor, which, in concert, may contribute to the development of hypertension in patients with insulin resistance [87]. There is also evidence that insulin resistance and hyperinsulinemia lead to SNS activation, and, as a result, the kidneys increase sodium reabsorption, the heart increases cardiac output, and arteries respond with vasoconstriction resulting in hypertension [88]. It has been recently discovered that adipocytes also produce aldosterone in response to ATII [89]. In this regard, the adipocyte may be considered a miniature renin-angiotensin-aldosterone system.

The article "A Comprehensive Review on Metabolic Syndrome" was retracted in 2019. Reasons: plagiarism; overlap with other authors' work.

### 5.5. Genetics

The great variations in the susceptibility and age of onset in individuals with a very similar risk profile suggest a major interaction between genetic and environmental factors [90]. It is recognized that some people who are not obese by traditional measures nevertheless are insulin-resistant and have abnormal levels of metabolic risk factors. Examples are seen in individuals with 2 diabetic parents or 1 parent and a first- or second-degree relative [91]; the same is true for many individuals of South Asian ethnicity [92]. Considerable individuals and ethnic variations also exist in the clinical pattern of metabolic risk factors in obese/insulin-resistant subjects [93]. It is likely that the expression of each metabolic risk factor falls partially under its own genetic control, which influences the response to different environmental exposures. For example, a variety of polymorphisms in genes affecting lipoprotein metabolism are associated with the worsening of dyslipidemia among obese people [94]. Similarly, a genetic predisposition to the defective insulin secretion when combined with insulin resistance can raise the plasma glucose to abnormal levels [95]. According to the* thrifty genotype hypothesis* proposed by Neel in 1962 [96], individuals living in a harsh environment with an unstable food supply would maximize their probability of survival if they could maximize a storage of surplus energy. Genetic selection would thus favour the energy-conserving genotypes in such environments. However, the selected genetic variations that were favoured during malnutrition would become unfavourable when nutrition improved. This hypothesis assumes that the common genetic variants of thrifty genes predispose to MetS. Another* thrifty phenotype hypothesis* was introduced by Hales and Barker in 1992 [97]. According to this hypothesis, babies who experienced an intrauterine malnutrition may have adapted to a poor nutrition by reducing energy expenditure and becoming “thrifty.” These metabolic adaptations are beneficial when individuals are poorly nourished during childhood and adult life; however, with an increased food intake, these adaptations are no longer beneficial and would lead to an increased risk of MetS in a later life. Support for this hypothesis comes from the observed associations of low birth weight with later development of insulin resistance and T2DM in several populations [98].

The article "A Comprehensive Review on Metabolic Syndrome" was retracted in 2019. Reasons: plagiarism; overlap with other authors' work.

### 5.6. Endothelial Function

It is characterized by an impaired endothelium-dependent vasodilatation, a reduced arterial compliance, and an accelerated process of atherosclerosis [107]. Various factors like oxidative stress, hyperglycemia, advanced glycation products, FFAs, inflammatory cytokines, or adipokines cause an inability of endothelium to serve its normal physiological and protective mechanisms. Hansson has shown that immune cells play an important role in all the stages of the atherosclerotic process [108]; in addition, a reduction in NO, a key regulator of endothelial homeostasis, and an increase in reactive oxygen species result in an endothelial dysfunction and a proatherogenic vascular bed [109].

### 5.7. Hypercoagulable State

A proinflammatory state is characterized by elevated circulating cytokines and acute-phase reactants (e.g., CRP). Further, a prothrombotic state signifies anomalies in the procoagulant factors, that is, an increase in fibrinogen, factor VII and factor VIII as well as the antifibrinolytic factor (PAI-1), platelet abrasions, and endothelial dysfunctions. Grundy [110] has shown that a fibrinogen, an acute-phase reactant protein like CRP, rises in response to a high-cytokine state. This shows that the prothrombotic and proinflammatory states may be metabolically interconnected.

### 5.8. Diet

A study by Aljada et al. has shown that a high dietary fat intake is associated with an oxidative stress and an activation of the proinflammatory transcription factor, that is, nuclear factor kappa-beta (NF*κ*B) [111]. In contrast, a diet rich in fruits and fibres has no inflammation-inducing capacity compared with a high-fat diet even if it has the same calories content [112].

### 5.9. Chronic Stress and Glucocorticoid (GC) Action

Chronic hypersecretion of stress mediators, such as cortisol, in individuals with a genetic predisposition exposed to a permissive environment, may lead to the visceral fat accumulation as a result of chronic hypercortisolism, low growth hormone secretion, and hypogonadism [113]. GCs increase the activities of enzymes involved in fatty acid synthesis and promote the secretion of lipoproteins [114]; induce the hepatic gluconeogenic pathway [115]; promote the differentiation of preadipocytes to adipocytes, which could lead to an increased body fat mass [116]; inhibit an insulin-stimulated amino acid uptake by adipocytes [117]; and increase lipolysis or lipid oxidation which leads to the peripheral insulin resistance [118]. A good correlation was observed between plasma cortisol levels, total urinary GC metabolites, and the number of features of the MetS among these patients. Both the secretion rate and the peripheral clearance of cortisol in these patients were positively correlated with the systolic blood pressure, and fasting glucose and insulin [119]. These hormonal alterations may lead to a reactive insulin hypersecretion, an increasing visceral obesity, and sarcopenia, resulting in dyslipidemia, hypertension, and T2DM [120].

The article "A Comprehensive Review on Metabolic Syndrome" was retracted in 2019. Reasons: plagiarism; overlap with other authors' work.

## 6. Treatment

MetS is a state of chronic low grade inflammation with the profound systemic effects (Table 3). Clinical identification and management of patients with the MetS are important to begin efforts to adequately implement the treatments to reduce their risk of subsequent diseases [121]. Effective preventive approaches include lifestyle changes, primarily weight loss, diet, and exercise, and the treatment comprises the appropriate use of pharmacological agents to reduce the specific risk factors. Pharmacological treatment should be considered for those whose risk factors are not adequately reduced with the preventive measures and lifestyle changes [122]. The clinical management of MetS is difficult because there is no recognized method to prevent or improve the whole syndrome, the background of which is essentially insulin resistance [15]. Thus, most physicians treat each component of MetS separately, laying a particular emphasis on those components that are easily amenable to the drug treatment. In fact, it is easier to prescribe a drug to lower blood pressure, blood glucose, or triglycerides rather than initiating a long-term strategy to change people's lifestyle (exercise more and eat better) in the hope that they will ultimately lose weight and tend to have a lower blood pressure, blood glucose, and triglycerides. For the treatment of risk factors of MetS, the physician should follow the current treatment guidelines of the National Cholesterol Education Programme (NCEP) [123], the seventh Joint National Commission (JNC-VII) for blood pressure treatment [124], the American Diabetes Association (ADA) [125], the American Heart Association (AHA) [20], and the National Institute of Health Obesity Initiative [126].

### 6.1. Risk Assessment

The goals of therapy are to reduce both a short-term and lifetime risk. The presence of the MetS* per se* indicates a higher lifetime risk. A practical approach to estimate absolute, short-term CHD/CVD risk in patients with the MetS without ASCVD or diabetes is to use the standard Framingham algorithm to estimate a 10-year risk of the coronary heart disease (CHD) [123]. The standard Framingham risk equations, which include cigarette smoking, blood pressure, total cholesterol, HDL-C, and age, capture most of the risk of CVD in patients with the syndrome. This equation triages patients into 3 risk categories based on a 10-year risk of CHD:* high risk* (10-year risk ≥20%),* moderately high risk* (10-year risk 10% to 20%), or* lower to moderate risk* (10-year risk ≤10%), while affected patients with ASCVD or diabetes are already in a high-risk category without the need for Framingham risk scoring.

The article "A Comprehensive Review on Metabolic Syndrome" was retracted in 2019. Reasons: plagiarism; overlap with other authors' work.

### 6.2. Lifestyle Modification

Lifestyle modification treatment should be delivered by a multidisciplinary approach (Table 4) and a team composed of physicians and nonphysician health professionals, such as dieticians or professionals with a master degree in exercise physiology, behavioural psychology, or health education [127]. Although lifestyle therapy may not modify any given risk factor as much as will a particular drug, its benefit lies in the fact that it produces a moderate reduction in all the metabolic risk factors [128].

### 6.3. Weight Reduction

Four therapies can be used for weight reduction: calorie restriction (e.g., 500 kcal/d deficit), increased physical activity, behavioural modification, and, in appropriate patients, FDA-approved weight-reducing drugs [128]. Several authors [20] recommend a weight loss goal of 10% reduction in body weight in the first six months to a year and continued weight loss thereafter until BMI is less than 25. While many patients find weight loss difficult to achieve, exercise and dietary changes that can lower blood pressure and improve lipid levels will further improve insulin resistance, even in the absence of weight loss [129]. A weight loss of as small as 5–10% of body weight can significantly reduce TGs and increases HDL-C [130]. Furthermore, both hypertensive individuals and individuals at risk of developing hypertension can see a significant reduction in the blood pressure with a modest weight loss [131]. Fasting blood glucose, insulin, and haemoglobin A1c can also be decreased with a modest weight loss [132]. During weight maintenance (i.e., energy balance), a regular exercise appears to play an important role in abdominal fat loss [133] and the prevention of weight regain in those who have successfully lost weight [134]. Persons who combine calorie restriction and exercise with behavioural modifications should expect to lose 5–10% of preintervention weight over a period of four to six months. This weight loss appears small to the patient but results in an improvement of many obesity related conditions including various abnormal components of the MetS and development of diabetes [135]. Both the Finnish Diabetes Prevention Study [136] and the US Diabetes Prevention Program (DPP) [137] showed that diet and exercise had a significant effect on reducing the progression from IGT to T2DM.

The article "A Comprehensive Review on Metabolic Syndrome" was retracted in 2019. Reasons: plagiarism; overlap with other authors' work.

### 6.4. Diet

The effective and healthful methods for the long-term weight loss are reduced-energy diets, consisting of a modest 500 to 1000 calories/day reduction. Sustained dietary changes may require a referral to a registered dietician to help implement the suggestions and ensure an adequate micronutrient intake (e.g., calcium, iron, and folate) while reducing calories. In the SUN (Seguimiento University of Navarra) prospective cohort study [138], a Mediterranean-style diet was inversely associated with the cumulative incidence of MetS. Adherence to the Mediterranean diet improves the physical and mental domains of health related quality of life (physical function, vitality, general physical health, emotional role, and self-perception of health) [139] and lowers the odds of LDL-C, postchallenge glucose values [140], TGs, and low HDL-C levels [141]. In the PREMIER study [142], the Dietary Approaches to Stop Hypertension (DASH) diet plus lifestyle interventions improved the metabolic parameters, particularly blood pressure. ATP III [123] recommended that the diet should contain 25% to 35% of calories as total fat for the individuals entering cholesterol management. If the fat content exceeds 35%, it is difficult to sustain the low intakes of saturated fat required to maintain a low LDL-C. On the other hand, if the fat content falls below 25%, TGs can rise and decline in HDL-C levels can be seen [143]; thus, a very low-fat diet may exacerbate an atherogenic dyslipidemia. A protein intake of 10–35% of total calorie intake is recommended by the Institute Of Medicine (IOM) for the general population with an exception of individuals with chronic kidney disease (CKD) who have markedly reduced glomerular filtration rate, where, an excess protein enhances phosphorus load, which can cause acidosis and worsen the insulin resistance [144]. Adherence may be enhanced by increasing the diet structure and limiting food choices, thereby reducing a temptation and the potential mistakes on calculating an energy intake [145]. A strategy to increase the diet structure is to provide patients with the meal plans, grocery lists, menus, and recipes. Support for this strategy is derived from a study showing that the provision of both low-calorie foods (free of charge or subsidized) and structured meal plans resulted in significantly greater weight loss than a diet with no additional structure [146]. Another effective strategy to increase dietary adherence is the meal replacements [147] which help to overcome some problems that occur while consuming the conventional food diets (i.e., underestimation of calorie intake, difficulties in estimating portion sizes, macronutrient composition, calorie content, and in recalling the consumed food). A clear positive association has been shown between sodium intake and blood pressure, with excessive sodium intake associated with hypertension [148]. Furthermore, a sodium restriction has also been associated with reduced CVD events [149] and congestive heart failure [150]. Guidelines therefore recommend that a daily sodium intake should be restricted to no more than 65–100 mmol [151]. In addition to sodium restriction, an increased potassium intake has also been shown to improve blood pressure, especially in the setting of high sodium intake [152]. Guidelines have recommended the intake of foods enriched with potassium, such as fruits and vegetables, with a goal of 90–120 mmol of potassium per day [151]. Incorporation of monounsaturated fatty acid (fat from plant source like olive oil, soybean oil, canola oil, safflower oil, peanut oil, peanuts, peanut butter, almond, and cashew nut) may be beneficial as it improves the atherogenic dyslipidemia. Similarly, n-3 polyunsaturated fatty acids (mainly from fish) have cardioprotective effect and it should constitute approximately 10% of total energy intake. Viscous (soluble) fibres (mainly in oat products, psyllium, and pectin) intake of 10–25 g/day also improves an atherogenic dyslipidemia [153]. Low glycemic index foods (i.e., those that are minimally processed) have been shown to improve the components of the MetS including hyperlipidemia and hyperglycemia [154], whereas, a higher glycemic index has been shown to be positively associated with the insulin resistance and MetS prevalence [155]. Therefore, a diet high in complex, unrefined carbohydrates with an emphasis on fibres (14 g/1000 calories consumed daily) and low in added sugars (≤25% of calorie intake) is recommended for individuals with or at risk of the MetS.

The article "A Comprehensive Review on Metabolic Syndrome" was retracted in 2019. Reasons: plagiarism; overlap with other authors' work.

### 6.5. Physical Activity

Current physical activity guidelines [156] recommend practical, regular, and moderate regimens for exercise. The standard exercise recommendation is a daily minimum of 30 minutes of moderate-intensity physical activity. However, a preference is given to 60 minutes of moderate-intensity brisk walking to be supplemented by other activities [157]. The latter includes multiple short (10 to 15 minutes) bouts of activity (walking breaks at work, gardening, or household work), using simple exercise equipment (e.g., treadmills), jogging, swimming, biking, golfing, team sports, and engaging in resistance training [158]; avoiding common sedentary activities in a leisure time (television watching and computer games) is also advised. Current AHA guidelines [156] call for a clinical assessment of the risk of the future ASCVD events before initiating a new exercise regimen. For high-risk patients (e.g., those with recent acute coronary syndromes or recent revascularization), physical activity should be carried out under the medical supervision. Clinicians should evaluate which type of activity is feasible for the patient, considering the barriers (e.g., arthritis and time constraints) that can prevent a successful increase in the physical activity. Accordingly, they should assist patients in developing a physical activity plan based on the initial assessment. However, any type of physical activity should be encouraged. Lifestyle activity should be increased slowly in intensity and duration (by 5 min/session/week), starting from a low-intensity exercise (<3 metabolic equivalent) in sedentary subjects, to avoid excessive fatigue, muscle pain, strains, or injuries [159]. Patients should be encouraged to register their baseline physical activity or to check their baseline number of steps by a pedometer. Whenever the brisk walking is chosen as the preferred activity, they should be instructed to add 500 steps at 3-day intervals to a target value of 10,000–12,000 steps/day [126]. Prescribing multiple short bouts (10 min each) rather than one long session may help the patients to accumulate more minutes of exercise. This 30 minutes of physical activity achieved in three 10-minute sessions is equivalent to the energy expenditure of 1500 kcal a week. The impact of exercise on insulin sensitivity is evident for 24 to 48 hours and disappears within three to five days. Thus, an individual would need to follow the AHA and American College of Sports Medicine recommendation to exercise at least 30 min/d most days of the week [160] for a continued benefit of exercise on insulin action. Physical training has been shown to reduce the skeletal muscle lipid levels and insulin resistance, regardless of BMI [161]. A combination of resistance and aerobic exercise is the best, but any activity is better than none, and patients who have been sedentary need to start with walking and gradually increase duration and intensity [162]. According to the Centre for Disease Control and Prevention (CDC) and the American College of Sports Medicine, physically inactive or sedentary subjects were defined as those who did not engage in at least 150 minutes of physical activities per week [163]. The odds of having the MetS were almost doubled in adults reporting no moderate or vigorous physical activity compared with those who engage in at least 150 min/wk [164]. Furthermore, Koplan and Dietz have shown that a regular exercise improves insulin sensitivity, decreases plasma TGs levels, and reduces cardiovascular morbidity and mortality [165].

The article "A Comprehensive Review on Metabolic Syndrome" was retracted in 2019. Reasons: plagiarism; overlap with other authors' work.

### 6.6. Behaviour Therapy

It has been designed to provide the patients with a set of principles and techniques to modify their eating and activity habits [145]. The emphasis in behavioural change should include the benefit of social support, stress management, the value of a regular exercise regimen, and an improvement in eating habits (e.g., setting goals, planning meals, reading labels, eating regular meals, reducing portion sizes, self-monitoring, and avoiding eating binges). Originally, the treatment was exclusively based on the learning theory (behaviourism). The theory postulates that the behaviours causing obesity (excess eating and low exercising) are largely learnt and therefore could be modified or relearnt. The theory further postulated that the positive changes in eating and exercising can be achieved by modifying the environmental cues (antecedents) and the reinforcements of these behaviours [166]. The intervention was later integrated with the cognitive strategies (e.g., problem solving and cognitive restructuring) and with the specific recommendations on diet and exercise [167]. Exercise promotion to decrease the chronic disease risk is also important in adults and the middle-aged since it can slow down the functional decline associated with ageing [168].

### 6.7. Pharmacological Approach

The National Institutes of Health guidelines for the treatment of obesity recommend a consideration of pharmaceutical therapy for weight loss for the individuals with a BMI of at least 30 kg/m^2^ or for those with a BMI of at least 27 kg/m^2^ and comorbidities associated with their excess weight. Pharmacological approaches to weight loss include two main classes: appetite suppressants and inhibitors of nutrient absorption. A single agent is generally recommended and an average weight loss ranges greatly from 5% to 10% of initial weight [169]. Appetite suppressants include phentermine derivatives and sibutramine. These agents are usually taken in the late morning and reduce appetite in the late afternoon and evening. Krejs reported that sibutramine-induced weight loss and weight maintenance lead to clinically relevant reductions in the risk factors associated with the syndrome [170]. Treatment with the drug decreases visceral fat, improves lipid levels, and decreases glycosylated haemoglobin and uric acid concentrations. Orlistat (an inhibitor of gastrointestinal lipase) is the only nutrient absorption inhibitor currently available. It prevents absorption of up to 30% of the fat consumed and must be taken at the time of consumption. Undesirable side effects such as flatulence and oil leakage in the stool often occur early in the course of treatment with this medication. In randomized clinical trials, orlistat in obese persons with T2DM at baseline led to an improved glycemic control and a weight reduction of 6% over 1 year versus 4% weight loss with placebo [171]. A recently published meta-analysis concerning the efficacy of pharmacological agents for obesity reported that an average weight loss was approximately four kilograms more than for placebo users and that no drug or class of drugs was clearly superior [172]. However, the major problem with these currently available antiobesity drugs is a relatively high rate of adverse side effects leading to a poor tolerance and compliance for the long-term use.

The article "A Comprehensive Review on Metabolic Syndrome" was retracted in 2019. Reasons: plagiarism; overlap with other authors' work.

### 6.8. Bariatric Surgery

Surgery is recommended for the individuals who do not respond to weight loss diet or medications, are extremely obese (BMI > 40 kg/m^2^), or if they have a BMI > 35 to 40 kg/m^2^ and one or more comorbid conditions [169]. Improvements in the metabolic profile have been documented presumably due to the redistribution of adiposity [174]. Bariatric surgery techniques using laparoscopic adjustable banding of stomach along with Roux-en-Y and other forms of gastric bypass are now favoured for the severe and morbid obesity [18]. It results in a weight loss of 25–30% and rapid normalization of glucose handling and blood pressure in patients with diabetes and hypertension [175] with 95% of patients being free of the syndrome one year after a surgery [18]. It has been found to be associated with the improvement and resolution of multiple comorbidities associated with obesity, including hypertension, T2DM, NAFLD, OSA, cardiopulmonary failure, CVD, arthritis, PCOS, dyslipidemia (exclusive of hypercholesterolemia), hyperuricemia, and infertility [175]. However, the long-term results are not available and recent reports of substantial mortality and morbidity of this procedure, especially in the elderly, have raised important safety issues for this procedure [176].

### 6.9. Dyslipidemia

The guidelines recommend that the LDL-C goals (Table 5) should be set at less than 130 mg/dL with the option of targeting less than 100 mg/dL in the moderately high-risk individuals. Target goals should be set at an LDL-C less than 100 mg/dL in the high-risk patients with the option of aiming for less than 70 mg/dL in the “very high-risk” patient [173]. The goal for the non-HDL-C is 30 mg/dL greater than LDL-C. In patients with an atherogenic dyslipidemia in whom the serum TGs levels are ≥200 mg/dL, non-HDL-C becomes the next target of treatment after the LDL-C goal is reached. If the TGs level is higher than 500 mg per dL, then lowering the TGs level to 500 mg per dL or less takes primacy over LDL-C lowering to prevent the development of acute pancreatitis. After LDL-C and non-HDL-C goals are achieved, a tertiary target is raising the HDL-C level. No goals for raising HDL-C levels are specified but HDL-C should be raised to the possible extent after attaining the goals for LDL-C and non-HDL-C [123].

The article "A Comprehensive Review on Metabolic Syndrome" was retracted in 2019. Reasons: plagiarism; overlap with other authors' work.

Statins are considered to be the most effective class of drugs for reducing the LDL-C concentrations due to their minimal drug-drug interactions and side effects [123]. Depending on the dose and the specific type of statin used, LDL-C reductions of 15 to 60 mg/dL are observed [177]. Statins increase HDL-C by 5–10%, with greater increases seen in individuals with lower HDL-C and elevated TGs, and reduce TGs concentrations by 7–30% primarily with moderate to high doses [178] and further decrease very low density lipoprotein (VLDL) levels by 39% [157]. Non-lipid-lowering or pleiotropic effects of statins have also been implicated in their beneficial effects on inflammation, endothelial function, and CVD events [179] and may therefore be beneficial for individuals with the MetS [180]. Statins also lower the incidence of MI or stroke by more than 33% in patients with coronary artery disease. Statins can also be safely combined with a fibrate, especially fenofibrate, and niacin to achieve the target levels of non-HDL-C, TGs, and HDL-C [7]. All statins had favourable effects on atherogenic dyslipidemia, with rosuvastatin generally having the greatest effect [181].

Niacin has favourable effects on essentially all of the abnormalities of the metabolic dyslipidemia. It is considered the most effective agent for raising HDL-C (15 to 35%) and increasing HDL particle size [182]. Niacin significantly lowers TGs (20 to 50%) and LDL-C (5–25%) [123]. Niacin also causes beneficial changes in the lipoprotein subclasses because it has been shown to reduce the proportion of small, dense LDL-C particles while increasing large, more buoyant LDL-C particles and larger HDL-C particles [183]. Combination therapy of a niacin and statin produces greater effects on the lipid levels than does an either agent given alone [184]. The primary limitations for the use of niacin include flushing (most often associated with immediate-release niacin) and hyperglycemia [185]. Therefore, if nicotinic acid is used in patients with impaired fasting glucose (IFG), impaired glucose tolerance (IGT), or diabetes, its dose should be kept relatively low (e.g., 1 to 2 g per day) and deserves careful monitoring for the worsening of hyperglycemia [186]. Niacin has the greatest effect on increasing HDL-C levels (15%–35%), with fibrates (6%–15%) and statins (3%–15%) having a more moderate effect [123].

The article "A Comprehensive Review on Metabolic Syndrome" was retracted in 2019. Reasons: plagiarism; overlap with other authors' work.

The two fibrates currently used clinically are gemfibrozil and fenofibrate, both of which can lower TGs by 25% to 30% with the greater reductions in individuals that are hypertriglyceridemic. Fibrates further increases HDL-C by 5–15% and reduces LDL-C by 0–30% [187]. Although fibrates reduce the plasma TGs and increase the HDL-C extent when used in patients with diabetes mellitus, there have been no studies specifically examining the effect of fibrates treatment in patients with the MetS [188]. The advantage of gemfibrozil is that it is lower in cost, but fenofibrate has a fewer drug interactions, especially when prescribed along with a statin. Several studies have reported an isolated severe myopathy occurring from the combination of a statin with gemfibrozil due to pharmacological interaction of statin glucuronidation and increase in the level of statins when used in conjunction [157]. ATP III has recommended the combination of fenofibrate and statin due to a very low risk of associated myopathy [7]. Although the treatment with statin/fibrate and statin/niacin has been reported to increase the risk of drug induced myopathy and rhabdomyolysis, such combination therapies are considered safe [189]. Low or intermediate doses of statins (10–40 mg/day) with fenofibrate (200 mg/day) or bezafibrate (400 mg/day) are considered effective and safe for the treatment of an atherogenic dyslipidemia [190]. Risk factors that predispose patients to myopathy caused by the above combinations include increased age, female sex, renal or liver disease, diabetes, hypothyroidism, debilitated status, surgery, trauma, excessive alcohol intake, heavy exercise, uncontrolled dose of niacin or fibrate, and use of additional medications (cyclosporine, protease inhibitors, or drugs metabolised through cytochrome P450) [191].

Bile acid sequestrants (BAS) and cholesterol absorption inhibitors (CAI) lower the LDL-C by decreasing the absorption of intestinal bile acids and cholesterol, respectively. BAS results in 15 to 30% reductions in LDL-C [192]. The only clinically available CAI, ezetimibe, has been shown to result in 15–25% reductions in LDL-C [193]. Although BAS and CAI are both effective as monotherapy, the greater benefits are obtained when used in combination with statins, an effect that may be due to their complementary mechanism of actions [194]. The study trial has shown that BAS and ezetimibe reduce the potential risk of major coronary events in patients with the MetS [195].

### 6.10. Hypertension

Categorical hypertension (BP ≥ 140/≥ 90 mm Hg) should be treated according to the USA JNC VII guidelines on the prevention, detection, evaluation, and treatment of the high blood pressure recommendations [124]. Antihypertensive drugs should be introduced at even lower blood pressures (≥130/≥80 mm Hg) in the patients with established diabetes. Mild elevations of blood pressure often can be effectively controlled with the lifestyle therapies. A simple 5% weight reduction in obese women lowered the systolic blood pressure by 7 mmHg and was associated with the decreased levels of angiotensinogen (−27%), renin (−43%), angiotensin-converting enzyme (−12%), aldosterone (−31%), and angiotensinogen expression in adipocytes (−20%) [196]. It is estimated that 5 mmHg reduction of systolic blood pressure across the general population would result in overall reductions of 14% in stroke mortality, 9% in CHD mortality, and 7% in all cause mortality [197]. However, if hypertension cannot be adequately controlled by lifestyle therapies, antihypertensive drugs usually are necessary to prevent the long-term adverse effects, for example, MI, stroke, and CKD [124]. It has been proposed that angiotensin converting enzyme (ACE) inhibitors or angiotensin receptor blockers (ARBs) should be the first-line classes of agents in the MetS, especially in the setting of diabetes or CKD [198]. ARBs may be used in those who cannot tolerate ACE inhibitors or as an alternative to ACE inhibitors in people who have a left ventricular dysfunction [199]. Certainly these classes of agents have been shown to be effective in reducing the incidence of albuminuria or progression of nephropathy in patients with diabetes [200]. Although a number of trials have shown that ACE inhibitors and ARBs may reduce the risk of diabetes [201], a more recent study designed to examine this issue directly found that the ACE inhibitor ramipril did not prevent the progression of diabetes in persons with IFG or IGT [202]. In general, treatment with these classes of drugs reduces the rate of new-onset diabetes as compared with the use of diuretic and/or *β*-blockers [203] but the long-term safety and efficacy of *β*-blockers and diuretics has been effectively demonstrated in many clinical trials, including the Antihypertensive and Lipid-Lowering treatment to prevent Heart Attack Trial (ALLHAT) that included >40,000 patients [204]. The ALLHAT showed that the treatment with a thiazide-type diuretic in patients with the MetS results in superior CVD outcomes compared to the treatment with calcium channel blockers, *β*-blockers, or ACE inhibitors despite the less favourable metabolic profile associated with the thiazide diuretics [205]. The ALLHAT and the United Kingdom Prospective Diabetes Study (UKPDS) have shown that agents such as thiazide diuretics and *β*-blockers lower the risk of CVD events even in the patients with diabetes [206]. These agents, however, have also been associated with an increased risk for diabetes [205, 206]. Certainly the majority of patients who need an antihypertensive therapy will likely need more than one agent for the proper blood pressure control [207].

The article "A Comprehensive Review on Metabolic Syndrome" was retracted in 2019. Reasons: plagiarism; overlap with other authors' work.

### 6.11. Insulin Resistance and Hyperglycemia

In MetS, patients with IFG (or IGT if assessed), weight reduction, increased physical activity, or both will delay (or prevent) the onset of T2DM [137]. In addition, metformin [137], thiazolidinediones [208], and acarbose [209] will lower the risk of T2DM in people with IFG or IGT. Metformin, which has a primary mechanism of action of reducing hepatic glucose production, has been shown to reduce the progression of diabetes from IGT by approximately 31% in the DPP, of which 53% had the MetS [137]. Incidence of the MetS was also reduced by 17% in the metformin-treated group of the DPP, which was driven primarily by improvements in WC and fasting glucose, whereas, intensive therapeutic lifestyle changes reduced this risk by 58% compared to placebo [210]. Other cardiac risk factors, however, did not improve with metformin to the same degree as with the intensive lifestyle intervention [211]. The study trial has suggested that metformin is in fact treating IGT and not necessarily “preventing” progression to T2DM in the long-term follow-up [212]. In the Study to Prevent Non-Insulin Dependent Diabetes Mellitus (STOP-NIDDM) trial, acarbose, a drug that affects carbohydrate absorption and is approved for the treatment of T2DM, was also shown to reduce the progression to T2DM in individuals with IGT [209]. This trial also showed that acarbose treatment was in fact associated with reduced CVD and hypertension [213]. The main limitation of the use of this agent is its poor patient tolerability. Pioglitazone has been shown to reduce the multiple components of MetS such as high blood pressure, high blood glucose, and TGs in addition to a decrease in urinary albumin/creatinine ratio [214]. It was concluded that pioglitazone may be useful in the prevention of cardiovascular events in high risk patients with T2DM although the usefulness of this approach in MetS or IGT subjects is not clear. However, no clinical trial evidence is yet available to document that the oral hypoglycemic agents will lessen the risk for cardiovascular events in MetS, IGT, or IFG except for a preliminary trial with acarbose [213].

### 6.12. Hypercoagulable State

Measurement of CRP is the most practical way to assess the presence of an inflammatory state. An elevated CRP (≥3 mg/L) is an emerging risk factor for CVD [123]. The AHA and CDC [215] recently issued guidelines for the measurement of CRP in the clinical practice. They suggested that such measurements can be made at the physician's discretion, but testing should be limited to the individuals assessed to be at an intermediate risk by Framingham scoring, that is, those whose 10-year risk for CHD is in the range of 10% to 20%. Several drugs used to treat the other metabolic risk factors have been reported to reduce the CRP levels (e.g., statins, nicotinic acid, fibrates, ACE inhibitors, and thiazolidinediones) [216]. However, these drugs cannot be recommended specifically to reduce a proinflammatory state independent of their indications for the other risk factors. Furthermore, The Justification for the Use of statins in Primary Prevention: an Intervention Trial Evaluating Rosuvastatin (JUPITER) trial [217] has emphasized an added benefit of statin in targeting the individuals with high CRP levels even in the presence of normal LDL. Low-dose aspirin is frequently recommended to the patients with MetS [218]; however, the use of aspirin in the primary prevention of CVD should remain as an “individual clinical judgment” [219]. Further, there is no evidence to indicate that the use of aspirin in low-risk groups (<6%) is beneficial, and the risk of haemorrhage outweighs the benefit in this category. Patients in the low intermediate risk group (6–10%) will need an individualized decision-making, whereas most patients in the conventional intermediate risk category (10–20%) should receive aspirin. Blaha et al. have advised that all older patients (≥65 years old) and patients at high Framingham risk with MetS should receive a low-dose aspirin in the absence of contraindications [220]. A recently published meta-analysis shows that aspirin significantly reduces the risk of first MI by a third, stroke by approximately one-third, and CVD by approximately one sixth [221].

The article "A Comprehensive Review on Metabolic Syndrome" was retracted in 2019. Reasons: plagiarism; overlap with other authors' work.

## 7. Conclusion

MetS is defined by a constellation of interconnected physiological, biochemical, clinical, and metabolic factors that directly increases the risk of atherosclerotic cardiovascular disease, type 2 diabetes mellitus, and all cause mortality. Insulin resistance, visceral adiposity, atherogenic dyslipidemia, endothelial dysfunction, genetic susceptibility, elevated blood pressure, hypercoagulable state, and chronic stress are the several factors which constitute the metabolic syndrome. Lifestyle modification remains the initial intervention of choice for this population. Modern lifestyle modification therapy combines specific recommendations on diet and exercise with behavioural strategies. Pharmacological treatment should be considered for those whose risk factors are not adequately reduced with lifestyle changes.

A realistic goal for overweight/obese persons is to reduce the body weight by >7% to 10% over a period of 6 to 12 months. Weight reduction should be combined with a daily minimum of 30 minutes of moderate-intensity physical activity. Nutritional therapy calls for a low intake of saturated and total fat intake; reduced consumption of simple sugars and high glycemic index foods; and increased intakes of fruits, vegetables, legumes, and whole grains. Statins can be combined with fibrates and niacin to achieve the target levels of LDL-C, triglycerides, and HDL-C. Further, the majority of patients who need an antihypertensive therapy will likely need more than one agent for the proper blood pressure control with ACEI/ARBs and beta blockers/Thiazides/CCBs as the first and second line agents, respectively. Metformin, thiazolidinediones, and acarbose will lower the risk for type 2 diabetes mellitus in people with IFG or IGT.

## Figures and Tables

**Figure 1:** Schematic presentation of MetS. (FFA: free fatty acid, ATII: angiotensin II, PAI-1: plasminogen activator inhibitor-1, RAAS: renin angiotensin aldosterone system, SNS: sympathetic nervous system.)

**Table 1:** Diagnostic criteria proposed for the clinical diagnosis of the MetS.

Clinical measures	WHO (1998) [5]	EGIR (1999) [6]	ATPIII (2001) [7]	AACE (2003) [8]	IDF (2005) [9]
Insulin resistance	IGT, IFG, T2DM, or lowered insulin Sensitivity^a^ **plus any 2 of the following**	Plasma insulin >75th percentile **plus any 2 of the following**	**None, but any 3 of the following 5 features**	IGT or IFG **plus any of thefollowing based on the clinical judgment**	None

Body weight	Men: waist-to-hip ratio >0.90; women: waist-to-hip ratio >0.85 and/or BMI > 30 kg/m^2^	WC ≥94 cm in men or ≥80 cm in women	WC ≥102 cm in men or ≥88 cm in women	BMI ≥ 25 kg/m^2^	Increased WC (population specific) **plus any 2 of the following**

Lipids	TGs ≥150 mg/dL and/or HDL-C <35 mg/dL in men or <39 mg/dL in women	TGs ≥150 mg/dL and/or HDL-C <39 mg/dL in men or women	TGs ≥150 mg/dL HDL-C <40 mg/dL in men or <50 mg/dL in women	TGs ≥150 mg/dL and HDL-C <40 mg/dL in men or <50 mg/dL in women	TGs ≥150 mg/dL or on TGs Rx. HDL-C <40 mg/dL in men or <50 mg/dL in women or on HDL-C Rx

Blood pressure	≥140/90 mm Hg	≥140/90 mm Hg or on hypertension Rx	≥130/85 mm Hg	≥130/85 mm Hg	≥130 mm Hg systolic or ≥85 mm Hg diastolic or on hypertension Rx

Glucose	IGT, IFG, or T2DM	IGT or IFG (but not diabetes)	>110 mg/dL (includes diabetes)	IGT or IFG (but not diabetes)	≥100 mg/dL (includes diabetes)^b^

Other	Microalbuminuria: Urinary excretion rate of >20 mg/min or albumin: creatinine ratio of >30 mg/g.			Other features of insulin resistance^c^	

^a^Insulin sensitivity measured under hyperinsulinemic euglycemic conditions, glucose uptake below lowest quartile for background population under investigation.

^b^In 2003, the American Diabetes Association (ADA) changed the criteria for IFG tolerance from >110 mg/dl to >100 mg/dl [10].

^c^Includes family history of type 2 diabetes mellitus, polycystic ovary syndrome, sedentary lifestyle, advancing age, and ethnic groups susceptible to type 2 diabetes mellitus.

The article "A Comprehensive Review on Metabolic Syndrome" was retracted in 2019. Reasons: plagiarism; overlap with other authors' work.

BMI: body mass index; HDL-C: high density lipoprotein cholesterol; IFG: impaired fasting glucose; IGT: impaired glucose tolerance; Rx: receiving treatment; TGs: triglycerides; T2DM: type 2 diabetes mellitus; WC: waist circumference.

**Table 2:** Gender and age-specific waist circumference cut-offs [1].

Country/ethnic group	Waist circumference cut-off	
	Male (cm)	Female (cm)
Europids In USA, the ATPIII values (102 cm males; 88 cm females) are likely to continue to be used for clinical purposes.	≥94	≥80
South Asians Based on a Chinese, Malay, and Asian-Indian population.	≥90	≥80
Chinese	≥90	≥80
Japanese	≥90	≥80
Ethnic South and Central Americans	Use South Asians recommendations until more specific data are available.	
Sub-Saharan Africans	Use European data until more specific data are available.	
Eastern Mediterranean and Middle East (Arabs) population	Use European data until more specific data are available.	

**Table 3:** Systemic effects of MetS.

Renal	Microalbuminuria, hypofiltration, hyperfiltration, glomerulomegaly, focal segmental glomerulosclerosis, and chronic kidney disease [99].
Hepatic	Increased serum transaminase, nonalcoholic steatohepatitis (NASH), nonalcoholic fatty liver disease (NAFLD), hepatic fibrosis, and cirrhosis [100].
Skin	Acanthosis nigricans, lichen planus, systemic lupus erythematosus, burn-induced insulin resistance, psoriasis, androgenetic alopecia, skin tags, skin cancer, and acne inversa [101].
Ocular	Nondiabetic retinopathy, age related cataract-nuclear, cortical, posterior subcapsular; central retinal artery occlusion, primary open angle glaucoma, oculomotor nerve palsy, and lower lid entropion [102].
Sleep	Obstructive sleep apnea (OSA) [103].
Reproductive system	Hypogonadism, polycystic ovarian syndrome (PCOS), and erectile dysfunction [104].
Cardiovascular system	Coronary heart disease (CHD), myocardial infarction (MI), and stroke [105].
Cancers	Breast, pancreas, and prostrate [106].

**Table 4:** Multidisciplinary approach to the MetS.

A: assessment	Calculate Framingham risk score: *high risk *(10-year risk ≥20%), *moderately high risk *(10-year risk 10% to 20%), or *lower to moderate risk *(10-year risk ≤10%). Make diagnosis of MetS using the diagnostic criteria.

A: aspirin	High risk: aspirin definitely beneficial. High-intermediate risk (10–20%): aspirin likely to be beneficial. Low-intermediate risk (6–10%): “individual clinical judgment”, depending on sex and risk of bleeding. Low risk (<6%): Risk of haemorrhage outweighs the benefits.

B: BP control	Initiate treatment: categorical hypertension (BP ≥ 140/≥90 mm Hg). Patients with established diabetes (≥130/≥80 mm Hg). ACEIs/ARBs first line agent may reduce incident diabetes mellitus. Beta-blockers and thiazides may have an adverse effect on impaired glucose tolerance but outweighed by the benefits of reaching BP goal and lowering the risk of CVD events.

C: cholesterol First target: LDL Second target: non-HDL Third target: HDL Fourth target: CRP	Statin to achieve LDL-C <100 mg/dL in high-risk, <130 mg/dL in intermediate-risk, and <160 mg/dL in low risk patients. Statin intensification, consider niacin and/or fibrates once statin maximized. Consider fibrates, especially for those with combined hypertriglyceridemia/low HDL-C. Consider further reduction in LDL-C with statin therapy to mitigate a risk of low HDL-C, consider niacin. Statin therapy for those with high sensitivity CRP (hsCRP) ≥3 mg/dL.

D: diabetes prevention/diet	Intensive lifestyle modification is the most important therapy. Weight reduction of 5–10% of preintervention weight over a period of four to six months. Sodium intake of <65–100 mmol/day with a goal of 90–120 mmol of potassium per day. Mediterranean diet: high consumption of fruits, vegetables, legumes, and grains, moderate alcohol intake, a moderate-to-low consumption of dairy products and meats/meat products, and a high monounsaturated- to-saturated fat ratio. DASH diet: rich in fruits, vegetables, and low-fat dairy products, and low in saturated and total fat intake. Consider low glycemic index food, complex unrefined carbohydrates, viscous soluble fibres, protein intake of 10–35% of total calorie intake and 25% to 35% of calories as total fat. Metformin is second line in delaying the onset of T2DM. Thiazolidinediones (Pioglitazones) and alpha-glucosidase inhibitors (Acarbose) have shown benefit in smaller studies and are therefore third line.

E: exercise	Daily moderate intensity activity of minimum 30 minutes for most days of the week. Recommend use of pedometer with goal >10,000 steps/day.

The article "A Comprehensive Review on Metabolic Syndrome" was retracted in 2019. Reasons: plagiarism; overlap with other authors' work.

**Table 5:** Goals for lowering LDL-C [173].

Risk category	LDL-C goals	Recommendations
Lower risk 0-1 major risk factor 10-yr risk <10%	<160 mg/dL	Lifestyle modifications Consider pharmacotherapy if LDL-C ≥190 mg/dL after lifestyle modifications

Moderate risk ≥2 major risk factors 10-yr risk <10%	<130 mg/dL	Lifestyle modifications Consider pharmacotherapy if LDL-C ≥160 mg/dL after lifestyle modifications

Moderately high risk ≥2 major risk factors 10-yr risk 10–20%	<130 mg/dL Optional <100 mg/dL	Lifestyle modifications Consider pharmacotherapy if LDL-C ≥130 mg/dL or optionally ≥100 mg/dL after lifestyle modifications

High risk CHD or CHD risk equivalents	<100 mg/dL Optional <70 mg/dL	Lifestyle modifications Consider pharmacotherapy if LDL-C ≥100 mg/dL or optionally ≥70 mg/dL after lifestyle modifications
